The article "Kukoamine A Improves Mycoplasma pneumoniae Pneumonia by Regulating miR-222-3p/Superoxide Dismutase 2" was retracted in 2023. Reasons: signs of a paper mill; compromised peer review; unreliable results or conclusions.

# Kukoamine A Improves *Mycoplasma pneumoniae* Pneumonia by Regulating miR-222-3p/Superoxide Dismutase 2

**DOI:** 10.1155/2022/2064013

**Published:** 2022-06-21

**Authors:** Xiu-Xiu Liu, Ming-Jing Wang, Qian-Na Kan, Cui Li, Zhen Xiao, Yong-Hong Jiang, Wen Li, Xiao Li, Zhi-Yan Jiang

**Affiliations:** ^1^Department of Pediatrics, Longhua Hospital Affiliated to Shanghai University of Traditional Chinese Medicine, Shanghai 200032, China; ^2^Institute of Respiratory Diseases, Longhua Hospital Affiliated to Shanghai University of Traditional Chinese Medicine, Shanghai 200032, China

## Abstract

*Mycoplasma pneumoniae* pneumonia (MPP) represents a common respiratory disease in children patients. Kukoamine A (KuA) is a spermine alkaloid found in the Chinese herb *Cortex Lycii radices*, which has a variety of pharmacological properties. However, no study has been reported on the role of KuA in MPP. Exosomes, a type of lipid bilayer-enclosed extracellular vesicles, can be delivered to the target cells, where they regulate function and physiology. With the use of human alveolar basal epithelial cells (HABECs) as an *in vitro* model, in this study, we sought to characterize the changes in levels of superoxide dismutase 2 (SOD2) and proinflammatory cytokines including IL-6 and TNF-*α* in HABECs in response to exosomes, which were isolated from peripheral blood serum of MPP patients. We found that, compared to normal, MPP patients exhibited a significant up-regulated miR-222-3p. Further, exosomal miR-222-3p downregulated SOD2 activity but promoted nuclear NF-*κ*B activity and expression of IL-6 and TNF-*α* in HABECs, ultimately leading to an oxidative stress condition. Interestingly, such stimulating effects were attenuated by the pretreatment of KuA. This study suggests a critical role possessed by KuA in MPP by regulating the miR-222-3p/SOD2 axis, which represents a promising strategy for the treatment of MPP.

## 1. Introduction

*Mycoplasma pneumoniae* pneumonia (MPP) is a common respiratory disease in pediatric patients, which results from an infection of *Mycoplasma pneumoniae* (*M. pneumoniae*). *M. pneumoniae* accounts for approximately 40% of community acquired pneumonia while about 18% of cases usually require hospitalizations [1–3]. *M. pneumoniae* respiratory diseases usually present similar clinical features to those observed with other atypical pathogens, for example, *Chlamydia pneumoniae*, and other various respiratory viruses and bacteria [4–6]. However, the etiology and pathogenesis of MPP remain largely unknown. A number of studies have shown that excessive host immune reactions may have partially contributed to the development of MMP, resulting in activation of lymphocytes including T helper (Th)1 and Th17 cells [7, 8]. While this activation and differentiation of Th1 and Th17 is tightly regulated by costimulatory molecules expressed on antigen presenting cells [9]. Moreover, the levels of various types of proinflammatory cytokines including IL-6 and TNF-*α* are also increased in MPP [10]. With regard to treatment, MPP could be self-limiting. However, clinicians routinely treat this disease with antibiotics. Interestingly, Qingfei Tongluo formula (QTF), a traditional Chinese medicine formula, can be an effective therapeutic approach for clinical treatment of MPP [11]. At molecular levels, we found that a treatment of QTF led to effective inhibition of activation of phosphorylation of c-Jun N-terminal kinase (JNK), extracellular signal-regulated kinase (ERK), and nuclear factor-*κ*B (NF-*κ*B) signaling pathways in the MPP mouse model [12]. Notably, Kukoamine A (KuA) constitutes a major active ingredient in the QTF formula. KuA is a spermine alkaloid present in traditional Chinese medicine *Cortex Lycii radices* and has various pharmacological properties [13]. However, there are no studies on the role of KuA in MPP.

The article "Kukoamine A Improves Mycoplasma pneumoniae Pneumonia by Regulating miR-222-3p/Superoxide Dismutase 2" was retracted in 2023. Reasons: signs of a paper mill; compromised peer review; unreliable results or conclusions.

Through their metabolites, exotoxin and exotoxin-like toxic substances of *M. pneumoniae* can cause remarkable toxin-like effects [14]. *M. pneumoniae* can infiltrate bronchial mucous membranes to release hydrogen peroxide, thereby causing swelling and necrosis of bronchial epithelial cells; consequently, leading to a reduced microvilli movement and deformation of structure for dissemination of lymphocytes and other immune cells [15]. Superoxide dismutase 2 (SOD2) and catalases are antioxidant enzymes and play a crucial role in controlling reactive oxygen species production, and the latter is a natural by-product of oxidative phosphorylation. ROS damages multiple components of the cell and thereby disturbs diverse biological processes, such as cell metabolism, aging, and death [16]. The other prevailing virulence factors influencing the pathogenesis of *M. pneumoniae* also include accumulated hydrogen peroxide within the host cells and deleterious effects by superoxides on host cellular ultrastructure [17]. In addition, *M. pneumoniae*-produced ions can effectively impede activities of SOD and catalases in the host cells. As such, host cells become more susceptible to toxic oxygen, thus leading to mitochondrial enlargement and impaired cilia movement in lung epithelium [18].

An increasing body of evidence supports that noncoding RNAs including microRNAs (miRNAs) play important roles in regulation of varied types of physiological processes including cell differentiation and proliferation and apoptosis [19]. Indeed, Chu and colleagues have recently profiled miRNAs in the peripheral blood of pediatric MPP patients and found that 26 miRNAs were differentially regulated between MPP and normal controls [20]. Their further *in vivo* study revealed that miR-222-3p, an upregulated miRNA in MPP patients, could be a meaningful indicator for diagnosis and prognosis of MPP [18].

The article "Kukoamine A Improves Mycoplasma pneumoniae Pneumonia by Regulating miR-222-3p/Superoxide Dismutase 2" was retracted in 2023. Reasons: signs of a paper mill; compromised peer review; unreliable results or conclusions.

Over the past decades, evidence has begun to accumulate that exosomes can be transported to the target cells, where they are capable of regulating function and physiology. Exosomes are lipid bilayer-enclosed extracellular vesicles that encompass constituents including protein, DNA, and RNA of the cells that generate them, with a size range of 40 to 160 nm in diameter with an endosomal origin [21, 22]. Such discoveries suggest that exosomes circulating in patients' blood may also play a role in regulating the physiology and function of lung cells and tissues in MPP. Indeed, through employing miRNA-sequencing (miRNA-seq) on peripheral blood serum exosomes from pneumoniae patients caused by human adenovirus, Huang et al. found that four miRNAs can distinguish pneumoniae patients from heathy controls, suggesting these miRNAs may contribute to the pathogenesis of this virus-induced pneumonia [23].

In the present study, using human alveolar basal epithelial cells (HABECs) as an *in vitro* model, we focused on characterizing the changes in levels of SOD2 and proinflammatory cytokines including IL-6 and TNF-*α* in HABECs, in response to exosomes, which were isolated from peripheral blood serum of MPP patients.

## 2. Materials and Methods

### 2.1. Medicine Information

Kukoamine A (KuA) was purchased from the company (75288-96-9, MedChemExpress (MCE), New Jersey, USA) and dissolved in DMSO.

### 2.2. Cell Culture

The human type-II alveolar epithelial (A549) cells were obtained from American Type Culture Collection (ATCC) and cultured in DMEM medium (Hyclone, SH30243.01; Logan, UT, USA) added with 10% fetal bovine serum (FBS; GIBCO, 16000-044; Carlsbad, CA, USA) and 1% penicillin-streptomycin (Solarbio, P1400, Beijing, China) and incubated in an incubator at 37°C with 5% CO_2_.

### 2.3. Plasmid Construction and Cell Transfection

The open reading frame sequences of SOD2 (NM_000636.4) were amplified with primers harboring Hind III/EcoR I restriction sites and ligated into pCDNA3.1 (+) to overexpress SOD2: SOD2-F: 5′-CCCAAGCTTATGTTGAGCCGGGCAGTG-3′ (Hind III) SOD2-R: 5′-CGGAATTCTTACTTTTTGCAAGCCATGTATC-3′ (EcoR I).

### 2.4. Cell Transfection

When in the logarithmic growth phase, A549 cell transfection was performed as recently described [24]. Briefly, A549 cells were trypsinized and counted to 1 × 10^6^ cells/ml suspension, and then, 2 ml of suspension was inoculated into 6-well plates for overnight culture at 37°C in a 5% CO_2_ incubator. When grown to 60-70% confluency, the cells were transfected with WT + NC, WT + inhibitor, WT + mimic, Mut + NC, Mut + inhibitor, Mut + mimic, or control, vector, and oeSOD2 by Lipo2000 (11668-019, Invitrogen). After 24 hours of transfection, serum-free transfer solution was instead of complete medium to culture for 48 hours. The sequences of miR-222-3p mimics and miR-222-3p inhibitor are 5′-AGCUACAUCUGGCUACUGGGU-3′ and 5′-ACCCAGUAGCCAGAUGUAGCU-3′, respectively. Nonspecific sequences are 5′-CAGUACUUUUGUGUAGUACAA-3′. miR-222-3p mimics and inhibitor were obtained from GenePharma (Shanghai, China).

The article "Kukoamine A Improves Mycoplasma pneumoniae Pneumonia by Regulating miR-222-3p/Superoxide Dismutase 2" was retracted in 2023. Reasons: signs of a paper mill; compromised peer review; unreliable results or conclusions.

### 2.5. Clinical Specimens

Patients' blood was prepared to collect exosomes as recently described [25]. All serum specimens (MPP patients: *n* = 10; healthy: *n* = 10) were stored at -80°C and further used for exosomes isolation. The protocol for the present study was approved by the Ethics Committee of Longhua Hospital Affiliated to Shanghai University of Traditional Chinese Medicine (Shanghai, China), and it conforms to the provisions of the Declaration of Helsinki in 1995. All participants have provided their written informed consent to participate in the study.

### 2.6. Isolation and Identification of Serum Exosomes

This procedure was performed as recently described [25]. Briefly, serum exosomes were individually extracted from the healthy (*n* = 10) and patients (*n* = 10) with MPP with 10,000 × g for 30 min at 4°C. Supernatants were then transferred to 5 mL ultrahigh speed centrifugal tubes (supplemented with 1 × PBS) and centrifuged twice at 17,000 g for another 2 h at 4°C, after which the supernatants were removed. The supernatants were then centrifuged again under the same conditions. The pellets were resuspended in the corresponding 1 × PBS, filtered with a 0.22 *μ*m filter, and then the exosomes were quantified using a BCA protein quantification kit, and then aliquoted and stored at -80°C for further analysis. Serum exosomes were identified by Western blot with the use of antibodies of anti-CD9 (Ab92726), anti-CD63 (Ab271286), and anti-CD81 (Ab109201) supplied from Abcam (Cambridge, England).

### 2.7. Fluorescent Labeling of Exosomes

Serum exosomes were labeled with PKH-67 Exosomes Green Fluorescent Dye (Umibio, USA) as recently described [24]. In brief, preparation of PKH67 dyeing working solution: at room temperature, the “PKH67 linker” was mixed with “Diluent C” at a ratio of 1 : 9 in the dark. Exosomes staining: exosomes were stained at room temperature by PKH67 for 4 h in the dark and visualized under a fluorescent microscope (Nikon, Japan).

The article "Kukoamine A Improves Mycoplasma pneumoniae Pneumonia by Regulating miR-222-3p/Superoxide Dismutase 2" was retracted in 2023. Reasons: signs of a paper mill; compromised peer review; unreliable results or conclusions.

### 2.8. Real Time-Quantitative PCR (RT-qPCR)

RT-qPCR was used to measure mRNA levels as previously described [26]. RNA samples were isolated using TRIZOL reagent and then reverse transcribed to cDNA using the RevertAid First Strand cDNA Synthesis Kit (Fermentas, Hanover, MD, USA), followed by amplified with the SYBR Green qPCR Master Mixes (#K0223, Thermo Fisher, Rockford, IL, USA) according to the manufacturers' instructions. The relative mRNA levels were estimated using the 2^-△△Ct^ method after normalized to GAPDH. The primer sequences (forward or F/reverse or R) were listed in Table 1.

### 2.9. Western Blot Analysis

Western blot assay was performed as recently described [26]. The lysates were separated by electrophoresis. Interest proteins were transferred to polyvinylidene fluoride (PVDF) membrane and blocked with 5% nonfat milk. Then, the bands were incubated with optimally diluted primary antibodies and HRP-labeled (antimouse and antirabbit) second antibodies sequentially. Protein expression was assessed with a chemiluminescent imaging system (Tanon 5200, Shanghai, China). Anti-CD9 (Ab92726, 1 : 1000), anti-CD63 (Ab271286, 1 : 2000), anti-CD81 (Ab109201, 1 : 700), and anti-SOD2 (Ab13534,1 : 2000) from Abcam (Cambridge, England), and anti-NF-*κ*B (#8242, 1 : 1000), anti-H3 (#4499, 1 : 1000), and anti-GAPDH (#5174, 1 : 2000) from CST (Boston, USA) served as primary antibodies.

### 2.10. ELISA Assay

The levels of IL-6 and TNF-*α* in supernatants were determined using an ELISA kit (X-Y Biotechnology, Shanghai, China) according to the manufacturer's instructions.

### 2.11. Luciferase Reporter Assays

All plasmids were constructed as recently detailed [24]. The sequence of SOD2 (NM_000636.4) promoter was amplified by PCR and placed into a pGL3-enhancer plasmid containing the firefly luciferase gene. SOD2 3′-UTR was inserted into pGL3-promoter vector to construct pGL3-promoter-wtSOD2. According to hsa-miR-222-3p and SOD2 3′-UTR binding site, the site-directed mutation SOD2 3′-UTR was inserted into pGL3-promoter vector to construct pGL3-promoter-mutSOD2. Cultured cells were cotransfected directly with the pGL3-promoter-wtSOD2 and the pRL-TK-Renilla reporter, or pGL3-promoter-mutSOD2 and the pRL-TK-Renilla reporter. After 6 h of transfection, cells were divided to treat with WT + NC, WT + inhibitor, WT + mimic, Mut + NC, Mut + inhibitor, and Mut + mimic. After 24 h, the dual-luciferase assay was conducted with Dual-Promoter Luciferase Assay Kit (Promega, USA).

### 2.12. Statistical Analysis

GraphPad Prism 7.0 software (San Diego, CA, USA) was used for statistical analysis. Each experiment was repeated at a minimum of three times. Data was shown in mean ± standard deviation (SD). One-way analysis of variance (ANOVA) was applied to analyze the differences of multiple groups. *P* < 0.05 was statistically significant.

The article "Kukoamine A Improves Mycoplasma pneumoniae Pneumonia by Regulating miR-222-3p/Superoxide Dismutase 2" was retracted in 2023. Reasons: signs of a paper mill; compromised peer review; unreliable results or conclusions.

## 3. Results

### 3.1. Serum Exosomes of MPP Patients Induce Inflammation in A549 Human Alveolar Basal Epithelial Cells

To study the role of serum exosomes from MPP patients, exosomes were isolated from the serum of healthy controls (normal control-exo) and MPP patients (MPP patients-exo) using ultrahigh-speed centrifugation. The purity was validated by transmission electron microscope (Supplementary Figure 1A) and characterized by the measurement of exosomes surface markers CD9, CD63, and CD81 (Supplementary Figure 1B). PKH-67 staining revealed that exosomes were endocytosed by A549 cells (Supplementary Figure 1C). All these results suggested that exosomes were successfully isolated and ready for further analysis.

Next, the effects of isolated serum exosomes on proinflammatory cytokines including IL-6 and TNF-*α* have been analysed. As shown in Figures 1(a) and 1(b), treatment of A549 cells with MPP patients' serum exosomes led to a significant increase of levels of IL-6 and TNF-*α* in supernatant, which was remarkably reversed by the addition of KuA in a dose-dependent manner. KuA possesses potent antihypertensive, antioxidant, and anti-inflammatory effects [27]. In our recent study, we also found that KuA constitutes a major active ingredient in QTF formula that has remarkably ameliorative effects on MPP in a mouse model [12].

Furthermore, Figures 1(c) and 1(d) showed that MPP exosomal treatment significantly inhibited SOD2 mRNA levels and resulted in increased expression of NF-*κ*B, while such a trend of decreased expression of SOD2 and increased level of NF-*κ*B can be reversed by KuA in a dose-dependent manner.

Taken together, these results suggest that MPP patients' serum exosomes can potently induce inflammation in human alveolar basal epithelial cells, and SOD2/NF-*κ*B pathway may be involved in this process.

### 3.2. miR-222-3p Is Highly Expressed in Exosomes and Induces Inflammation in Human Alveolar Basal Epithelial Cells

A previous study has shown that miR-222-3p was increased in MPP patients' serum [20]. Here, we hypothesized that such an increase in serum was attributed to the increased abundance of exosomes in serum, which was actually confirmed by RT-qPCR assay (Figure 2(a)).

In order to investigate the effects of miR-222-3p on levels of proinflammatory cytokines in A549 cells, first, we treated A549 cells with MPP serum exosomes as shown in Figure 2(b). The results suggested that the miR-222-3p level in A549 cells was augmented along with an increased incubation time with exosomes, while the parallel extracellular miR-222-3p levels at the corresponding incubation time points were significantly decreased (Supplementary Figure 2A), and there is no significant change in miR-222-3p level by A549 cells during the incubation (Supplementary Figure 2B). These findings suggest that A549 cells were highly capable of taking these serum exosomes. In Figures 2(c) and 2(d), SOD2 levels were reduced at both mRNA and protein levels along with extended exosomal exposure, which was coupled with increased nuclear NF-*κ*B activity in A549 cells (Figure 2(d)). In addition, IL-6 and TNF-*α* were also increased during exosomal exposure in a time-dependent manner (Figures 2(e) and 2(f)). Statistical test showed that the SOD2 level was negatively correlated with miR-222-3p level, whereas IL-6 and TNF-*α* levels were positively correlated with miR-222-3p level (Supplementary Figure 2C-2D).

The article "Kukoamine A Improves Mycoplasma pneumoniae Pneumonia by Regulating miR-222-3p/Superoxide Dismutase 2" was retracted in 2023. Reasons: signs of a paper mill; compromised peer review; unreliable results or conclusions.

Taken together, these data suggest that miR-222-3p may play an important role in serum exosomes from MPP patients, which can be delivered into A549 cells, triggering inflammation.

### 3.3. Mechanisms of miR-222-3p Repression of SOD2 Transcription in Human Alveolar Basal Epithelial Cells

Here, the molecular mechanisms underlying miR-222-3p-induced inhibition of SOD2 activity in A549 cells were further dissected. MicroRNA usually modulate gene expression through interaction with the 3′-UTR of the mRNA. And then 3′-UTR of wild-type (WT) and mutant SOD2 mRNA into luciferase reporter plasmid were constructed to test the effects of miR-222-3p on SOD2 expression. Figures 3(a)–3(c) revealed that transfection of miR-222-3p mimics caused a significant increase of miR-222-3p expression but significantly reduced endogenous mRNA and protein levels of SOD2, while miR-222-3p inhibitors had opposite effects. Furthermore, Figure 3(d) showed that miR-222-3p mimics significantly inhibited the activities of the SOD2 3′UTR. Next, a eukaryotic expression vector, allowing an ectopic expression of SOD2, was constructed, and the overexpression efficiency was detected (Supplementary Figure 3A-3B). Consistent with the above mentioned results, miR-222-3p mimics increased IL-6 and TNF-*α* levels. However, such effects were reversed by overexpressed SOD2 (Figures 3(e) and 3(f)). In addition, miR-222-3p-mediated elevation of nuclear NF-*κ*B activity was also reversed by an ectopic expression of SOD2 (Figure 3(g)). These findings further support that miR-222-3p promotes inflammation in A549 by inhibiting SOD2 activity.

### 3.4. KuA Attenuates miR-222-3p Mimic-Induced Inflammation by Targeting SOD2

We found that treatment of KuA did not alter miR-222-3p levels in A549 cells treated with MPP serum exosomes (Figure 4(a)). However, KuA was able to efficiently reverse MPP serum exosomes-mediated inhibition of SOD2 and increased nuclear NF-*κ*B activity in A549 cells (Figure 4(b)). Furthermore, treatment of KuA partly reversed miR-222-3p mimics increased IL-6 (Figure 4(c)) and TNF-*α* (Figure 4(d)) levels, as well as decreased SOD2 expression and elevation of nuclear NF-*κ*B activity (Figure 4(e)). Combined with the results showing that KuA had no discernable effects on levels of SOD1 and SOD3 in A549 cells (Supplementary Figure 4A-4B), it can be inferred that KuA partly attenuates miR-222-3p mimic-induced inflammation in A549 cells, which probably by targeting SOD2.

The article "Kukoamine A Improves Mycoplasma pneumoniae Pneumonia by Regulating miR-222-3p/Superoxide Dismutase 2" was retracted in 2023. Reasons: signs of a paper mill; compromised peer review; unreliable results or conclusions.

## 4. Discussion

*M. pneumoniae* represents a leading cause of community-acquired pneumonia and causes excessive inflammation that significantly exacerbates the severity of this disease. However, the mechanism and pathophysiology of such excessive inflammation are poorly understood. In this study, we found that MPP patients had a significantly increased expression of miR-222-3p in their peripheral blood serum exosomes as compared to the healthy counterparts.

Our investigation has found that upregulation of miR-222-3p in MMP has potential to decrease the activity of SOD2 and increase the expression of NF-*κ*B followed by upregulation of proinflammatory cytokines such as IL-6 and TNF-*α* in human alveolar basal epithelial cells and A549 cells and resulted in induction ROS generation. On the other hand, dose-dependent treatment of KuA partly reversed miR-222-3p mimic effects by inducing increased expression of proinflammatory cytokines, as well as elevation of nuclear NF-*κ*B activity. Our findings go hand in hand with a recent study showing that KuA-containing QTF formula alleviated MPP in mice [12, 28]. Studies have found that KuA protects against MDA-induced neurotoxicity by the induction of oxidative stress [29, 30]. Thus, it can be inferred that KuA alleviated MPP probably through regulating oxidative stress. This study provides a novel molecular route linking peripheral blood serum exosomes and induction of inflammation and oxidative stress in lung tissues of MPP patients.

Here, we first reported that miR-222-3p negatively regulates SOD2 but positively regulates proinflammatory cytokines in human alveolar basal epithelial cells A549. A number of studies on the functions of miR-222-3p in regulating gene expression in immune cells, such as macrophages, have mainly focused on its role in cancer [31, 32]. Recent studies by Lodge et al. suggest that miR-222-3p plays a role in the induction of viral infection through targeting CD4, a surface molecule on macrophages that actively participates in a variety of proinflammatory responses [33, 34]. Interestingly, few studies have suggested that MPP patients had a significantly increased abundance of miR-222-3p but a reduced level of CD4 mRNA in their peripheral blood monocytes [20]. Our study presented that MPP patients' serum exosomes can efficiently deliver miR-222-3p into human alveolar basal epithelial cells and thus suppress the SOD2 activity. Our study offers significant insights into the identification of novel targets through miR-222-3p in human alveolar basal epithelial cells and provides a novel mechanism involved in the pathogenesis of MPP.

The article "Kukoamine A Improves Mycoplasma pneumoniae Pneumonia by Regulating miR-222-3p/Superoxide Dismutase 2" was retracted in 2023. Reasons: signs of a paper mill; compromised peer review; unreliable results or conclusions.

This study highlights an important role of serum exosomes in the induction of inflammation and pathogenesis of MPP. Effective communication between various types of cells can be exemplified through exosomes. Indeed, the existence and possible role of extracellular vesicles in bacterial and viral infection have been well documented [35]. Exosomes released in response to stress conditions can be obviously distinguished by their contents including RNA and protein in comparison with those liberated from normal cells [36, 37]. The quality and amount of such extracellular vesicles also change with the physiological conditions of cells that release them. Furthermore, the release of extracellular vesicles can be prominently triggered by various stress factors, including bacterial infections. In consistent with these observations, our study supports that an increased secretion of exosomes and their contents in peripheral blood in response to *M. pneumoniae* infection can remarkably modulate the functions of effectors gene involved in the induction of inflammation, thus further contributing to a complicated pathophysiological condition in human lung tissues. The cellular origin of these miR-222-3p-contaning exosomes is unknown in this study, but could be a subject for future research.

In conclusion, this study supports a critical role of serum exosomal miR-222-3p in dysregulation of SOD2 activity and proinflammatory cytokines in human alveolar basal epithelial cells. Thus, blocking exosomes access to these cells could represent a promising strategy for the treatment of MPP.

## Figures and Tables

**Figure 1:** Serum exosomes of MPP patients induce inflammation in human alveolar basal epithelial cells A549. MPP serum exosomes (100 *μ*g/mL) were treated with A549 cells, followed by 24 h of treatment with KuA at different concentrations (0, 5, 10, and 20 *μ*M) as indicated. (a, b) ELISA assay for assessment expression of IL-6 (a) and TNF-*α* (b) in the cell supernatant. (c, d) RT-qPCR was used for assaying the mRNA expression levels of SOD2 (c) and NF-*κ*B (d) (3 repeats in each treatment group). ∗∗∗*P* < 0.001 vs. control (A549 cells without treatment); ^#^*P* < 0.05, ^##^*P* < 0.01, ^###^*P* < 0.001 vs. 100 *μ*g/ml_exo + 0 *μ*M_KuA; ^+^*P* < 0.05 vs. 100 *μ*g/ml_exo + 5 *μ*M_KuA; ^&^*P* < 0.05 vs. 100 *μ*g/ml_exo + 10 *μ*M_KuA.

The article "Kukoamine A Improves Mycoplasma pneumoniae Pneumonia by Regulating miR-222-3p/Superoxide Dismutase 2" was retracted in 2023. Reasons: signs of a paper mill; compromised peer review; unreliable results or conclusions.

**Figure 2:** miR-222-3p is highly expressed in exosomes and induces inflammation in human alveolar basal epithelial cells. (a) Exosomes extracted from serum samples from MPP patients and normal healthy controls, and then RT-qPCR was used for detecting the expression levels of miR-222-3p (*n* = 10; ∗∗∗*P* < 0.001 vs. control). (b)–(f) A549 cells were treated with MPP serum exosomes (100 *μ*g/mL) for 6, 12, and 24 h. (b, c) RT-qPCR was used to detect the mRNA expression levels of miR-222-3p (b) and SOD2 (c). (d) Western blot was used to detect the protein expression levels of SOD2 and NF-*κ*B. (e, f) at 6, 12, and 24 h, the expression of IL-6 (e) and TNF-*α* (f) in the cell supernatant was detected by ELISA. ∗*P* < 0.05, ∗∗*P* < 0.01, ∗∗∗*P* < 0.001 vs. 0 h; ^#^*P* < 0.05, ^##^*P* < 0.01 vs. 6 h; ^+^*P* < 0.05, ^++^*P* < 0.01 vs. 12 h.

**Figure 3:** Mechanisms of miR-222-3p repression of SOD2 transcription in human alveolar basal epithelial cells. (a)–(c) miR-222-3p inhibitors or mimics were transfected into A549 cells. (a) The miRNA expression of miR-222-3p was detected by RT-qPCR. ∗∗*P* < 0.01, ∗∗∗*P* < 0.001 vs. NC (negative control of mimics or inhibitors). (b, c) The mRNA (b) and protein (c) expression of the endogenous expression of SOD2 in A549 cells was detected by RT-qPCR. ∗∗*P* < 0.01, ∗∗∗*P* < 0.001 vs. NC. (d) Assay of luciferase activities in A549 cells transfected with wild-type (WT) or mutant (Mut) constructs along with miR-222-3p mimics or inhibitors as indicated. ∗∗*P* < 0.01, ∗∗∗*P* < 0.001 vs. WT + NC. (e)–(g) miR-222-3p mimics and SOD2 overexpression vectors were concomitantly or individually transfected into cells A549 cells. (e, f) ELISA for detecting the expression levels of IL-6 (e) and TNF-*α* (f) in the cell supernatant. (g) The protein expression of SOD2 and NF-*κ*B was detected by western blot. ∗∗*P* < 0.01, ∗∗∗*P* < 0.001 vs. NC; ^##^*P* < 0.01, ^###^*P* < 0.001 vs. mimic + vector.

**Figure 4:** KuA attenuates miR-222-3p mimic-induced inflammation by targeting SOD2. (a, b) A549 cells were treated with MPP serum exosomes (100 *μ*g/mL), followed by 24 h treatment of KuA at different concentrations (0, 5, 10, and 20 *μ*M) of as indicated. (a) The mRNA expression of miR-222-3p was detected by RT-qPCR. (b) The protein expression of SOD2 and NF-*κ*B (cytoplasm and nuclear) was detected by western blot. ∗∗∗*P* < 0.001 vs. control (A549 cells without treatment); ^#^*P* < 0.05, ^##^*P* < 0.01, ^###^*P* < 0.001 vs. 100 g/mL_exo + 0 *μ*M_KuA; ^+^*P* < 0.05, ^++^*P* < 0.01 vs. 100 g/mL_exo + 5 *μ*M_KuA; ^&^*P* < 0.05 vs. 100 g/mL_exo + 10 *μ*M_KuA. (c)–(e) A549 cells were treated with miR-222-3p mimics, followed by treatment of KuA at 10 *μ*M for 24 h. (c, d) ELISA to identify the levels of IL-6 (c) and TNF-*α* (d) in the cell supernatant. (e) The protein levels of SOD2 and NF-*κ*B (cytoplasm and nuclear) were examined by western blot. ∗∗*P* < 0.01, ∗∗∗*P* < 0.001 vs. control; ^#^*P* < 0.05, ^##^*P* < 0.01 vs. mimic + vehicle.

The article "Kukoamine A Improves Mycoplasma pneumoniae Pneumonia by Regulating miR-222-3p/Superoxide Dismutase 2" was retracted in 2023. Reasons: signs of a paper mill; compromised peer review; unreliable results or conclusions.

**Table 1:** The primer sequences (forward or F/reverse or R).

Name	Sequences
SOD1	Primer F 5′ CAGGGCATCATCAATTTC 3′ Primer R 5′ AGCCTGCTGTATTATCTC 3′
SOD2	Primer F 5′ ACAGGTTATGGTGGATTCAAAG 3′ Primer R 5′ AAACAATAGCCAGGGAAGTTAG 3′
SOD3	Primer F 5′ CCTCCATTTGTACCGAAAC 3′ Primer R 5′ GAAGATCGTCAGGTCAAAG 3′
NF-*κ*B	Primer F 5′ GCACAAGGAGACATGAAACAG 3′ Primer R 5′ CAGCCGGAAGGCATTATTAAG 3′
GAPDH	Primer F 5′ AATCCCATCACCATCTTC 3′ Primer R 5′ AGGCTGTTGTCATACTTC 3′
Hsa-miR-222-3p	Primer F 5′ GCGCGAGCTACATCTGGCTA 3′ Primer R 5′ AGTGCAGGGTCCGAGGTATT 3′
U6	Primer F 5′ CTCGCTTCGGCAGCACA 3′ Primer R 5′ AACGCTTCACGAATTTGCGT 3′

## Data Availability

The data that support the findings of this study are available from the corresponding author upon reasonable request.

## Abbreviation

MPP: Mycoplasma pneumoniae pneumonia
HABECs: Human alveolar basal epithelial cells
SOD2: Superoxide dismutase 2
KuA: Kukoamine A
QTF: Qingfei Tongluo formula
JNK: c-Jun N-terminal kinase
ERK: Extracellular signal-regulated kinase
NF-*κ*B: Nuclear factor-*κ*B.

## Supplementary Materials

Supplementary Materials Figure 1: clinical serum samples from children infected with *Mycoplasma pneumoniae* and normal healthy controls were collected. Then, serum exosomes were extracted by ultra-high speed centrifugation. (a) Transmission electron microscope analysis of contents and purity of exosomes. (b) Western blot to assess the abundances of exosomal markers CD81, CD63, and CD9. (c) Exosomes extracted from serum samples of MPP patients and normal healthy controls were incubated with A549 cells (2 × 10^5^ cells) for 4 h in the dark, and then uptake of PKH-67-labeled exosomes by A549 cells was performed. Figure 2: expression level of miR-222-3p in control and MMP patients has been detected. (a) A549 cells were treated with MPP serum exosomes (100 *μ*g/mL) for 6, 12, and 24 h, the parallel extracellular miR-222-3p levels were detected by RT-qPCR. (b) A549 cells were treated with MPP serum exosomes (100 *μ*g/mL) and RNA scavenger, then, RNA expression levels of miR-222-3p were detected by RT-qPCR. (c)–(e) The correlations between the miR-222-3p expression and expression levels of SOD2 (c), IL-6 (d), and TNF-*α* (e) in the exosomes extracted from serum samples from MPP patients (*n* = 10). Figure 3: SOD2 overexpression plasmid vectors were transfected into A549 cells. RT-qPCR (a) and Western blot (b) were used to discern SOD2 overexpression efficiency. ∗∗*P* < 0.01, ∗∗∗*P* < 0.001 vs. vector group. Figure 4: expression level MMPP serum exosomes after coincubation with A549 cell line have been detected followed by in control and MMP patients have been detected KuA treatment. (a, b) RT-qPCR was used to detect the abundances of SOD1 and SOD3. ∗∗*P* < 0.01, control group. ^#^*P* < 0.05 vs. 0 group.

The article "Kukoamine A Improves Mycoplasma pneumoniae Pneumonia by Regulating miR-222-3p/Superoxide Dismutase 2" was retracted in 2023. Reasons: signs of a paper mill; compromised peer review; unreliable results or conclusions.

## References

[1] Yan C., Sun H., Zhao H. (2016). Latest surveillance data on Mycoplasma pneumoniae infections in children, suggesting a new epidemic occurring in Beijing. *Journal of Clinical Microbiology*.

[2] Ferwerda A., Moll H. A., de Groot R. (2001). Respiratory tract infections by Mycoplasma pneumoniae in children: a review of diagnostic and therapeutic measures. *European Journal of Pediatrics*.

[3] Kashyap S., Sarkar M. (2010). Mycoplasma pneumonia: clinical features and management. *Lung India*.

[4] Becker A., Kannan T. R., Taylor A. B. (2015). Structure of CARDS toxin, a unique ADP-ribosylating and vacuolating cytotoxin from Mycoplasma pneumoniae. *Proceedings of the National Academy of Sciences of the United States of America*.

[5] Hu J., Chen C., Ou G. (2017). Nrf2 regulates the inflammatory response, including heme oxygenase-1 induction, by Mycoplasma pneumoniae lipid-associated membrane proteins in THP-1 cells. *Pathogens and Disease*.

[6] Somarajan S. R., Kannan T. R., Baseman J. B. (2010). Mycoplasma pneumoniae Mpn133 is a cytotoxic nuclease with a glutamic acid-, lysine- and serine-rich region essential for binding and internalization but not enzymatic activity. *Cellular Microbiology*.

[7] Guo L., Liu F., Lu M. P., Zheng Q., Chen Z. M. (2015). Increased T cell activation in BALF from children with Mycoplasma pneumoniae pneumonia. *Pediatric Pulmonology*.

[8] Kurata S., Osaki T., Yonezawa H., Arae K., Taguchi H., Kamiya S. (2014). Role of IL-17A and IL-10 in the antigen induced inflammation model by Mycoplasma pneumoniae. *BMC Microbiology*.

[9] Wen J., Wang H., Dong T. (2019). STAT3-induced upregulation of lncRNA ABHD11-AS1 promotes tumour progression in papillary thyroid carcinoma by regulating miR-1301-3p/STAT3 axis and PI3K/AKT signalling pathway. *Cell Proliferation*.

[10] Chen Z. R., Zhang G. B., Wang Y. Q. (2013). Soluble B7-H3 elevations in hospitalized children with _Mycoplasma pneumoniae_ pneumonia. *Diagnostic Microbiology and Infectious Disease*.

The article "Kukoamine A Improves Mycoplasma pneumoniae Pneumonia by Regulating miR-222-3p/Superoxide Dismutase 2" was retracted in 2023. Reasons: signs of a paper mill; compromised peer review; unreliable results or conclusions.

[11] Jiang Z. Y., Xiao Z., Jiang Y. H., Liu X. X. (2019). Effect of Qingfei Tongluo decoction on TCM syndrome score and serum inflammatory factors in children with Mycoplasma pneumoniae pneumonia. *World Science and Technology-Modernization of Traditional Chinese Medicine*.

[12] Jiang Y. H., Yu J. E., Guo A. H. (2016). Ameliorative effects of Qingfei Tongluo formula on experimental Mycoplasmal pneumonia in mice. *Journal of Natural Medicines*.

[13] Li G., Zhou F., Chen Y., Zhang W., Wang N. (2017). Kukoamine A attenuates insulin resistance and fatty liver through downregulation of Srebp-1c. *Biomedicine & Pharmacotherapy*.

[14] McDermott A. J., Taylor B. M., Bernstein K. M. (2013). Toxic epidermal necrolysis from suspected Mycoplasma pneumoniae infection. *Military Medicine*.

[15] Grosshennig S., Schmidl S. R., Schmeisky G., Busse J., Stulke J. (2013). Implication of glycerol and phospholipid transporters in Mycoplasma pneumoniae growth and virulence. *Infection and Immunity*.

[16] Han L., Wang H., Li L. (2017). Melatonin protects against maternal obesity-associated oxidative stress and meiotic defects in oocytes via the SIRT3-SOD2-dependent pathway. *Journal of Pineal Research*.

[17] Maenpuen S., Watthaisong P., Supon P. (2015). Kinetic mechanism of l–*α*–glycerophosphate oxidase from Mycoplasma pneumoniae. *The FEBS Journal*.

[18] Kariya C., Chu H. W., Huang J., Leitner H., Martin R. J., Day B. J. (2008). Mycoplasma pneumoniae infection and environmental tobacco smoke inhibit lung glutathione adaptive responses and increase oxidative stress. *Infection and Immunity*.

[19] Patil V. S., Zhou R., Rana T. M. (2014). Gene regulation by non-coding RNAs. *Critical Reviews in Biochemistry and Molecular Biology*.

[20] Chu C., Lei X., Li Y. (2019). High expression of miR-222-3p in children with Mycoplasma pneumoniae pneumonia. *Italian Journal of Pediatrics*.

[21] Zhang Y., Liu Y., Liu H., Tang W. H. (2019). Exosomes: biogenesis, biologic function and clinical potential. *Cell & Bioscience*.

[22] Johnstone R. M. (2006). Exosomes biological significance: a concise review. *Blood Cells, Molecules & Diseases*.

[23] Huang F., Bai J., Zhang J. (2019). Identification of potential diagnostic biomarkers for pneumonia caused by adenovirus infection in children by screening serum exosomal microRNAs. *Molecular Medicine Reports*.

[24] Hong Y., Sun Y., Rong X., Li D., Lu Y., Ji Y. (2020). Exosomes from adipose-derived stem cells attenuate UVB-induced apoptosis, ROS, and the Ca^2+^ level in HLEC cells. *Experimental Cell Research*.

[25] Qin D., Yang W., Pan Z., Zhang Y., Li X., Lakshmanan S. (2020). Differential proteomics analysis of serum exosomein burn patients. *Saudi Journal of Biological Sciences*.

The article "Kukoamine A Improves Mycoplasma pneumoniae Pneumonia by Regulating miR-222-3p/Superoxide Dismutase 2" was retracted in 2023. Reasons: signs of a paper mill; compromised peer review; unreliable results or conclusions.

[26] Zhou Q., Xiao Z., Zhou R. (2019). Ubiquitin-specific protease 3 targets TRAF6 for deubiquitination and suppresses IL-1*β* induced chondrocyte apoptosis. *Biochemical and Biophysical Research Communications*.

[27] Hu X. L., Niu Y. X., Zhang Q. (2015). Neuroprotective effects of Kukoamine B against hydrogen peroxide-induced apoptosis and potential mechanisms in SH-SY5Y cells. *Environmental Toxicology and Pharmacology*.

[28] Xiao Z., Jiang Y., Gao X. (2017). Comparison of the ameliorative effects of Qingfei Tongluo formula and azithromycin on Mycoplasma pneumoniae pneumonia. *Journal of Natural Medicines*.

[29] Yang Y., Gao L., Niu Y. (2020). Kukoamine A protects against NMDA-induced neurotoxicity accompanied with down-regulation of GluN2B-containing NMDA receptors and phosphorylation of PI3K/Akt/GSK-3*β* signaling pathway in cultured primary cortical neurons. *Neurochemical Research*.

[30] Hu X. L., Gao L. Y., Niu Y. X. (2015). Neuroprotection by Kukoamine A against oxidative stress may involve N-methyl- d-aspartate receptors. *Biochimica et Biophysica Acta*.

[31] Li Y., Zhao L., Shi B. (2015). Functions of miR-146a and miR-222 in tumor-associated macrophages in breast cancer. *Scientific Reports*.

[32] Ying X., Wu Q., Wu X. (2016). Epithelial ovarian cancer-secreted exosomal miR-222-3p induces polarization of tumor-associated macrophages. *Oncotarget*.

[33] Lodge R., Ferreira Barbosa J. A., Lombard-Vadnais F. (2017). Host microRNAs-221 and -222 inhibit HIV-1 entry in macrophages by targeting the CD4 viral receptor. *Cell Reports*.

[34] Lodge R., Gilmore J. C., Ferreira Barbosa J. A., Lombard-Vadnais F., Cohen E. A. (2018). Regulation of CD4 receptor and HIV-1 entry by microRNAs-221 and -222 during differentiation of THP-1 cells. *Viruses*.

[35] Zhang W., Jiang X., Bao J., Wang Y., Liu H., Tang L. (2018). Exosomes in pathogen infections: a bridge to deliver molecules and link functions. *Frontiers in Immunology*.

[36] Eldh M., Ekström K., Valadi H. (2010). Exosomes communicate protective messages during oxidative stress; possible role of exosomal shuttle RNA. *PLoS One*.

[37] de Jong O. G., Verhaar M. C., Chen Y. (2012). Cellular stress conditions are reflected in the protein and RNA content of endothelial cell-derived exosomes. *Journal of Extracellular Vesicles*.

